# An Investigation into the Correlation of Intestinal Flora with Obesity and Gestational Diabetes Mellitus

**DOI:** 10.1155/2022/5677073

**Published:** 2022-07-16

**Authors:** Zhiying Song, Shumin Li, Rongqin Li

**Affiliations:** ^1^Shanxi Provincial Children's Hospital (Shanxi Provincial Maternal and Child Health Care Hospital) Obstetrics Department, 030000, China; ^2^Graduate Student of Shanxi Medical University, 030000, China

## Abstract

**Method:**

Thirty-two pregnant women aged 25-35 who were hospitalized in Shanxi Maternal and Child Health Hospital from January 2019 to December 2019 were included for evaluation, including 15 normal pregnant women (NG_NO group), 6 pregnant women with GDM alone (G_NO group), and 7 pregnant women with overweight alone (NG_O group). Stools were collected from pregnant women at 24 and 37 weeks of gestation and newborns' first meconium. The v3-v4 variable region of the gut flora 16s rRNA was double-ended sequenced and bioinformatically analyzed using the Illumina MiSeq PE300 sequencing platform.

**Results:**

In the third trimester of pregnancy, there were significant differences in the composition of intestinal flora between the simple overweight group, simple GDM group, and normal pregnant group. From the second trimester to the third trimester, there was no significant change in the relative distribution of intestinal flora at the phyla classification level in normal pregnant women. The relative distribution of intestinal flora at the phylum level of newborns was significantly different from that of their mothers. The characteristic intestinal microbes of newborns in simple GDM group were g_Diaphorobacter, while the simple recombinant neonates were Nocardiaceae (f_Nocardioidaceae). In addition, the results showed significant differences in intestinal flora among the normal pregnant women group, simple GDM group, simple overweight group, and GDM overweight group. The results of *β* diversity analysis showed a significant difference in intestinal microflora species composition structure between the simple overweight group and the normal pregnant group in the second trimester of pregnancy. The species composition structure of intestinal flora was similar between the simple GDM group and the normal pregnant group. In the third trimester of pregnancy, there was no significant difference in the *β* diversity index among the groups, and the composition and structure of intestinal flora were similar. There were significant differences in the composition structure (*β* diversity) of intestinal flora between pregnant women and their newborns in each group (*P* < 0.05). Correlation analysis showed that the blood glucose values of oral glucose tolerance test (OGTT)_1 h and OGTT_2 h were positively correlated with Bacteroides (Bacteroides) and negatively correlated with Proteus (Prevotella), prepregnancy BMI was negatively correlated with Bacteroides, and weight gain during pregnancy was negatively correlated with Vibrio (Desulfovibrio) in Proteus. The birth weight of newborns was positively correlated with Actinomycetes (Actinomyces), Bacteroides (Faecalibacterium), and microbacilli (Dialister) and negatively correlated with Rolston (Ralstonia).

**Conclusion:**

Gut microbiota is strongly linked to obesity and gestational diabetes.

## 1. Introduction

Pregnant women who are overweight and obese are more likely to develop pregnancy complications such as gestational diabetes mellitus and gestational hypertension, resulting in a significantly higher incidence of adverse pregnancy outcomes. In recent years, the incidence of overweight and obesity has increased year by year, which seriously impacts the health of mothers and babies [1]. Changes in the abundance and diversity of intestinal flora species have been reported to be associated with the development of metabolic diseases such as obesity and diabetes mellitus [1].

Gestational diabetes mellitus (GDM) is a clinical syndrome in which abnormal glucose metabolism occurs or is first detected during pregnancy [2]. Epidemiological studies have shown that pregnant women with GDM have a significantly higher risk of developing complications (such as pregnancy-induced hypertension, premature rupture of membranes, infection, amniotic fluid, and postpartum hemorrhage) than normal pregnant women who are more likely to develop type 2 diabetes. In addition, prolonged intrauterine hyperglycemia environment significantly increases the risk of complications such as fetal miscarriage, neonatal hypoglycemia, fetal malformations, and macrosomia [3]. Many risk factors can contribute to the development of GDM, including a body mass index (BMI) of ≥25 kg/m^2^ before pregnancy, excessive weight gain during pregnancy, advanced age (>35 years), family history of diabetes, history of GDM, history of polycystic ovary syndrome, history of multiple abortions, and poor lifestyle habits [4]. In recent years, with the improvement of living standards, the generalization of delayed birth, and the full implementation of the two-child policy, the proportion of pregnant women of advanced age and the incidence of obesity and GDM have all increased significantly. The incidence of GDM in China is 17.5%-18%, which is a serious threat to the near- and long-term health of mothers and children [5]. The causes and pathogenesis of GDM are not fully understood, but the current findings suggest that it is similar to the pathogenesis of type 2 diabetes. In recent years, with the widespread use of 16S rRNA high-throughput sequencing technology and the development of proteomics and metabolomics, more and more studies have found that changes in the abundance and diversity of the intestinal flora play a crucial role in the development of GDM [6] and that maternal overweight may affect the early development of the offspring by influencing the neonatal intestinal flora [7].

The intestinal tract contains about 1013 to 1014 bacterial groups and is the largest microbial community in the human body [8]. The intestinal flora of the normal population is ranked in order of abundance by the phylum thick-walled bacteria, the phylum Bacteroides, the phylum Aspergillus, and the phylum Actinomycetes [9]. The gut microbiota can be divided into beneficial, harmful, and conditionally pathogenic bacteria according to their relationship to host health. Beneficial bacteria include bifidobacteria and lactobacillus. Harmful bacteria include Aspergillus, Pseudomonas, and Clostridium aeruginosa, while conditional pathogenic bacteria refer to bacteria that are harmful to the human body under certain conditions, such as Enterococcus and Escherichia coli. The gut microbiota can be interdependently adjusted to keep the richness and diversity of the microbiota in a state of dynamic balance, but the gut microbiota can also be dysregulated due to changes in the body's endocrine status, immune function, age, diet, and environment, leading to obesity, metabolic diseases such as diabetes, development of cardiovascular disease, inflammatory bowel disease, or psychiatric disease [10].

The approach to studying gut microbes has broadly gone through 3 stages culture-dependent methods, non-culture-dependent traditional molecular biology methods, to high-throughput sequencing methods. Traditional isolation and culture techniques are time-consuming and limited in the number of strains cultured, making it difficult to identify genetic diversity in samples. Sequencing-based high-throughput genomics techniques allow for highly sensitive and accurate quantification of gut microbes, obtaining information covering the entire microbial community. Bacterial 16S rRNA genes are characterized by conserved and variable regions spaced apart, with the variable regions being strain-specific, and it is now generally accepted that the sequences of the V3-V4 regions can represent all the results obtained by sequencing the 16S regions, so the taxonomic characteristics of each bacterium can be obtained by analyzing the sequences of the V3-V4 variable regions [11]. High-throughput sequencing-dependent histology technology enables taxonomic identification and precise quantification of mixed strains in complex samples by combining the advantages of high-throughput with the strain identification advantages of 16S rRNA genes [12].

In this study, we used 16S rRNA high-throughput sequencing technology to sequence the flora in fresh faces of pregnant women with GDM and overweight and used bioinformatics software to analyze the changes in the abundance and diversity of the flora in order to find out the relationship between the intestinal microbiota and GDM and overweight and to develop new ideas for the prevention and treatment of GDM and overweight in the future.

## 2. Method

### 2.1. Study Subjects

Pregnant women aged 25-35 years old who had their delivery and hospitalization at Shanxi Maternal and Child Health Hospital from January 2019 to December 2019 were enrolled. Our investigation was divided into two subresearch, including the research on overweight pregnant women and GDM pregnant women. There were no statistically significant differences in age, week of delivery, neonatal birth weight, and oral glucose tolerance test (OGTT) 2 h glucose values between the four groups. All patients completed the study, and none dropped out of the study halfway through.

#### 2.1.1. Overweight Pregnant Women

Exclusion criteria were as follows: history of gastrointestinal tumors, surgery, previous gastrointestinal disease, and gestational diabetes. Diagnostic criteria for overweight are as follows: BMI cut-off values established by WTO were used: overweight: 25 kg/m^2^ ≤ BMI < 28 kg/m^2^; normal BMI range: 18.5 to 24.9 kg/m^2^ [13]. According to the prepregnancy BMI, there were 20 cases in the normal BMI group and 20 cases in the overweight group. The first stool in the morning at 24 and 37 weeks of gestation was collected from each group of pregnant women, respectively. All pregnant women gave their informed consent, and the hospital ethics committee approved the project.

#### 2.1.2. GDM Pregnant Women

There were no abnormalities in blood routine, blood biochemistry, stool routine, and occult blood test except for diabetes detection index. Prepregnancy BMI was assessed, and a glucose tolerance test was performed at 24 weeks of pregnancy. Fifteen normal pregnant women (NG_NO group), 6 pregnant women with GDM alone (G_NO group), 7 pregnant women with overweight alone (NG_O group), and 4 pregnant women with overweight GDM (G_O group) were selected. All pregnant women gave their informed consent, and the hospital ethics committee approved the project.

Exclusion criteria were as follows: (1) type 1 diabetes; (2) gastrointestinal tumors and previous gastrointestinal surgery; (3) previous major bowel resection; (4) previous gastrointestinal disorders; (5) infections of the gastrointestinal, respiratory, and urinary tracts; (6) antibiotics within the last 2 months; (7) probiotics, laxatives, and antidiarrhea medication within the last 2 weeks; (8) hypertensive disorders of pregnancy and pregnancy with thyroid dysfunction; (9) pregnancy with hepatitis; (10) pregnancy with intrahepatic biliary depression; (11) heart disease combined with pregnancy; (12) cervical insufficiency; (13) in vitro fertilization; (14) premature rupture of membranes; and (15) anxiety and depression.

### 2.2. Diagnostic Criteria of Overweight and GDM

#### 2.2.1. Diagnostic Criteria for Overweight

The World Health Organization (WHO) body mass index (BMI) cut-off values are used: BMI = weight (kg)/height (m)^2^; normal BMI range: 18.5-24.9 kg/m^2^; overweight: 25 ≤ BMI < 28 kg/m^2^; obese: BMI ≥ 28 kg/m^2^ [13].

#### 2.2.2. Diagnostic Criteria of GDM

The “Guidelines for the Diagnosis and Management of Gestational Combined Diabetes Mellitus” was published by the Chinese Society of Obstetrics and Gynecology [14]. 75 g glucose tolerance test was performed at 24-28 weeks of gestation (fasting for at least 8 hours before the test, sitting still, and abstaining from smoking during the test after taking the glucose), with fasting and 1- and 2-hour glucose values of 5.1 mmol/l, 10.0 mmol/l, and 8.5 mmol/l, respectively. GDM will be diagnosed if any of these values are met or exceeded.

### 2.3. Main Experimental Reagents and Instruments

The details of the main experimental reagents and instruments applied in this research are exhibited in Tables 1 and 2.

### 2.4. Experimental Method

#### 2.4.1. Collection of Specimens

The collection method is as follows: pregnant women retained their own stools at 24 and 37 weeks of gestation using sterile EP tubes and were delivered to Shanxi Children's Hospital within 2 h and stored at -80°C in a refrigerator for backup. Due to force majeure factors, some pregnant women have changed their maternity check-ups and delivery hospitals, resulting in the first collection of fetal feces at 37 weeks of gestation and after the birth of their newborn not being completed (Table 3).

#### 2.4.2. DNA Extraction and Testing

DNA extraction was performed according to the instructions of the E.Z.N.A.® Soil Kit (Omega Bio-Tek, Norcross, GA, U.S.). 3.0 *μ*l of the extracted DNA sample was taken, and the concentration of the extracted DNA sample was measured using NanoDrop 2000. 1% agarose gel electrophoresis (voltage: 5 V/cm; time: 20 min) was used to detect the integrity of the sample DNA.

#### 2.4.3. PCR Amplification of 16s rRNA V3-V4 Variable Region

The primer profiles required for the experiments are listed in Table 4. The PCR test was performed using TransGen AP221-02 (TransStart FastPfu DNA Polymerase, 20 *μ*l reaction system, Table 5). The PCR amplification reaction procedure is shown in Table 6. The PCR instrument was ABI GeneAmp® Model 9700. PERMANOVA analysis based on Bray Curtis distance are listed in Table 7.

#### 2.4.4. Illumina MiSeq Sequencing

The PCR product was recovered using a 2% agarose gel, purified using the AxyPrep DNA Gel Extraction Kit (Axygen Biosciences, Union City, CA, USA), and eluted with Tris-HCl, and 3 *μ*l of PCR product was assayed using 2% agarose electrophoresis. Quantification was carried out using QuantiFluor™-ST (Promega, USA). The purified amplified fragments were then used to construct a PE 2∗300 library according to the Illumina MiSeq platform standard protocol (steps to construct the library: ligating the “Y” junction → using magnetic beads to screen for self-associated fragments → using PCR amplification to enrich the library template → denaturing with sodium hydroxide to produce (single-stranded DNA fragments). Finally, double-end sequencing was performed using Illumina's MiSeq PE300 platform.

### 2.5. Bioinformatics Analysis

Bacteria that differed in abundance between samples were identified using LEfSe analysis. Analysis of*α*-diversity and*β*-diversity was performed using the QIIME2 core-diversity plug-in.

### 2.6. Statistical Analysis

For general clinical data, data were analyzed using mean ± standard deviation (*x* ± *s*) and *t*-test using SPSS 22.0 statistical software. ANOVA for comparison of means between groups was used, and SNK test for comparison between two groups, with *P* < 0.05 indicating a statistically significant difference.

In the bioinformatics analysis, bacteria with differences in relative abundance between samples were identified using LEfSe analysis, and whether there were significant differences in the alpha diversity index between sample subgroups was compared using the Wilcoxon test, and whether there were significant differences in microbial composition between sample subgroups was compared using the PERMANOVA method, with *P* < 0.05 indicating a statistically significant difference.

## 3. Result

### 3.1. Comparison of General and Clinical Information of Pregnant Women in the Four Groups

The prepregnancy BMI of the normal BMI group was less than that of the overweight group, and the difference was statistically significant (*P* < 0.05). The GDM group gained less weight during pregnancy than the non-GDM group, and the difference was statistically significant (*P* < 0.05). The OGTT fasting glucose and OGTT 2 h glucose values of the GDM group were greater than those of the non-GDM group, and the difference was statistically significant (*P* < 0.05). The NG_O group (overweight group alone) and G_O group (GDM superreconstituted) had slightly higher birth weight than the NG_NO group (normal pregnant group), but the difference was not statistically significant (*P* > 0.05).

### 3.2. Analysis of the Species Composition of the Intestinal Flora

In this study, 79 fecal specimens were double-ended sequenced using the Illumina MiSeq platform. All raw sequences from all samples were quality controlled, denoised (corrected for sequencing errors), spliced, using the DADA2 plug-in in QIIME2 software to form OTUs, also known as signature sequences. The average number of sequences per specimen was 3536. OTUs were artificially assigned to a taxonomic unit (phylum, phylum, order, family, genus, and species) to facilitate analysis in phylogenetic or population genetic studies. Each OTU was usually regarded as a microbial species. Based on the absolute abundance of OTUs and annotation information, the number of sequences in each sample at each of the seven taxonomic levels (kingdom, phylum, class, order, family, genus, and species) as a proportion of the total number of sequences can be used to assess the species annotation resolution (proportion of annotations to genus/species) of a sample. The higher the percentage of annotation to genus/species, the better the OTU annotation of the sample (Figure 1).

### 3.3. Relative Distribution of Gut Flora Phylum Classification Levels between Groups

At midpregnancy (24 weeks), there was no significant difference in the relative distribution of the gut flora at the phylum level between the NG_NO group (normal pregnant women group), G_NO group (GDM-only group), NG_O group (super-recombinant alone), and G_O group (GDM super-recombinant). The thick-walled phylum was predominant (about 70%), followed by the phylum Bacteroides (about 13%), the phylum Actinobacteria (about 10%), and the phylum Aspergillus (about 5%) (see Figure 2(a)).

There was a significant difference in the composition of the intestinal flora between the overreconstituted GDM group and normal pregnant women at late pregnancy (37 weeks). Compared to the normal pregnant women group, the G_NO group (GDM-only group) showed an increase in the proportion of the phylum Bacteroides and a decrease in the proportion of the thick-walled phylum; the NG_O group (super-recombinant-only group) showed an increase in the proportion of the phylum Actinobacteria and a decrease in the proportion of the thick-walled phylum.

It can be seen that from mid- to late pregnancy, there was no significant change in the relative distribution of gut flora at the phylum classification level in the NG_NO group (normal pregnant women group). The proportion of the bacteriophage phylum increased, and the proportion of the thick-walled phylum decreased in the G_NO group (GDM-only group). Additionally, the proportion of the Actinomycetes phylum increased and the proportion of the thick-walled phylum decreased in the NG_O group (super-recombinant-only group) (see Figures 2(a) and 2(b)).

There was no significant difference in the relative distribution of gut flora at the phylum level between neonates in the G_NO group (GDM-only group), NG_O group (super-recombinant-only), and NG_NO group (normal pregnant group) in Figure 2(c). It can be seen that the relative distribution of intestinal flora at the phylum level in neonates was significantly different from that of their mothers. In neonates, the phylum Aspergillus was predominant (about 75%), followed by the thick-walled phylum and Actinomycetes, while their mothers are predominantly thick-walled (see Figures 2(a)–2(c)).

### 3.4. Analysis of the Significance of OTU Differences between Groups

The LDA bar graphs for LEfSe analysis of gut flora in pregnant women at 24 weeks gestation, 37 weeks gestation, and newborns, respectively, were shown. Each horizontal bar in the graph represents a species, and the length of the bar corresponds to the LDA value, with higher LDA values resulting in greater differences. The color of the bar corresponds to which subgroup of microorganisms was characteristic of that species, with characteristic microorganisms (LDA values > 2) indicating relatively high abundance in the corresponding subgroup (see Figures 3–5). Cladogram plots of the LEfSe analysis of the gut flora of pregnant women at 24- and 37-weeks' gestation and of newborns are represented in Figure 6.

The LEfSe analysis of the midpregnancy gut flora of each group of pregnant women showed that the characteristic gut microorganisms in the G_NO group (GDM-only group) at 24 weeks were the order o_Desulfovibrionales, f_Desulfovibrionaceae, c_ Deltaproteobacteria, and g_Anaerostipes; the characteristic intestinal microorganism in the G_O group (GDM super-recombinant) at 24 weeks was g_Lactobacillus. The characteristic intestinal microorganism in the NG_O group (simple superrecombinant) at 24 weeks was p_Verrucomicrobia, c_Verrucomicrobiae, o_Verrucomicrobiales, f_Verrucomicrobiaceae, and g_Akkermansia. The pregnancy group at 24 weeks had characteristic intestinal microorganisms of the genus Ruminococcus (g_Ruminococcus) (see Figure 3).

LEfSe analysis of the gut flora of each group of pregnant women in late pregnancy showed that the characteristic gut microorganisms in the G_O group (GDM superreconstituted) at 37 weeks were the genus Eubacterium (g_Eubacterium), the genus Conidium (g_Pyramidobacter), and the family Dethiosulfovibrionaceae (f_Dethiosulfovibrionaceae). The NG_O group (superrecombinant only) at 37 weeks showed characteristic gut microorganisms of Enterobacteriaceae (f_Enterobacteriaceae) and Enterobacteriaceae (o_Enterobacteriales).

LEfSe analysis of the intestinal flora of the neonates in each group showed that the characteristic intestinal microorganisms of the neonates in the G_NO group (GDM-only group) were the genus g_Diaphorobacter. The f_Nocardioidaceae were the characteristic intestinal microorganisms of the neonates in the NG_O group (GDM-only superreconstituted). The f_Nocardioidaceae was also the characteristic intestinal microorganisms of the neonates in the G_O group (GDM superreconstituted). The characteristic intestinal microorganisms of the G_O group (GDM superreconstituted) neonates are displayed in Figure 5.

### 3.5. Analysis of Shared Species between Groups

The OTU Venn diagrams for each group of pregnant women at 24 weeks showed (Figure 6(a)) that the number of OTUs shared between the four groups was a small proportion of the total number of OTUs in each group, indicating that the similarity between the four groups was not significant. The OTU Venn diagram for each group at 37 weeks (Figure 6(b)) showed an increase in the number of shared OUTs between the four groups at 37 weeks compared to 24 weeks, showing a slight decrease in the group differences in gut flora between the groups as the gestational weeks increased.

The OTU Venn diagram for each group (Figure 6(c)) showed that the total OTU count of the gut flora of neonates born to pregnant women in the NG_NO group was significantly higher than that of the G_NO and NG_O groups. The neonates were also significantly richer in intestinal flora than those born to diabetic and hyperrearranged pregnant women.

### 3.6. Analysis of the Significance of Differences in Beta Diversity of Intestinal Microorganisms

The PERMANOVA method was used to compare whether there was a significant difference in microbial composition structure between different subgroups of individual samples. The box plot of PERMANOVA analysis is shown in Figure 7 based on Bray Curtis distance between the different subgroups. In this study, a cross-sectional comparison of the groups of pregnant women at 24 weeks revealed a greater index of beta diversity between the NG_O group (superreconstituted only) and the NG_NO group (normal pregnant group), with a significant difference in species composition structure between the two groups (*P* < 0.05). In a longitudinal comparison, the composition of the intestinal flora was similar between the G_NO group (GDM only), the NG_O group (superrearranged only), and the NG_NO group (normal pregnant women) at 24 weeks and 37 weeks, but the difference in the composition of the intestinal flora between the pregnant women and their newborns was significant (*P* < 0.05).

### 3.7. Correlation Statistical Analysis

Correlation heat maps can be used to analyze whether environmental factors or clinical phenotypes are significantly correlated with microbial communities or species and then to calculate Spearman's correlation coefficients between environmental factors and microbial species. In this study, OGTT_1 h and OGTT_2 h blood glucose values were found to be significantly positively correlated with Bacteroides and negatively correlated with Prevotella. Fasting blood glucose values were not significantly correlated with intestinal flora. Prepregnancy BMI was negatively correlated with Bacteroides. Pregnancy weight gain was negatively correlated with Desulfovibrio in the phylum Aspergillus. The newborn birth weight was significantly positively correlated with Actinomyces, Faecalibacterium, and Dialister but negatively correlated with Ralstonia (see Figure 8).

## 4. Discussion

In recent years, more and more studies have shown that intestinal flora is closely related to the occurrence of overweight and GDM. In this paper, we used 16S rRNA sequencing technology to sequence the intestinal flora of normal pregnant women, overweight, and GDM pregnant women at different stages of pregnancy (mid- and late trimester) and their newborns.

In this study, the relative abundance of intestinal flora at the phylum level did not differ significantly from mid- to late pregnancy in normal pregnant women, with the thick-walled phylum predominating, followed by the phylum Bacteroides, the phylum Actinomycetes, and the phylum Aspergillus. Koren et al. found that the composition of the intestinal flora was similar to the nonpregnant state in early gestation and varied significantly in late gestation, with a significant decrease in the proportions of the thick-walled phylum and the phylum Bacteroides and an increase in the proportions of the phylum Actinobacteria and the phylum Aspergillus and a decreasing trend in the alpha diversity and an increasing trend in the beta diversity of maternal intestinal microorganisms from early to late gestation, which was different from the results of this study [15]. Differences in sample size, geographic location, antibiotic use, and dietary habits may account for differences in findings on gut microbiota changes in healthy pregnant women from early to late pregnancy.

The relative abundance of intestinal flora in the midpregnancy simple supergroup, the simple GDM group, the GDM supergroup, and the normal pregnant group did not differ significantly at the phylum classification level, but there were differential OTUs between the groups. The microorganisms with higher abundance in the midpregnancy simple GDM group were Vibrio desulfovibrionales (o_Desulfovibrionales), Vibrio desulfovibrionaceae (f_Desulfovibrionaceae), *δ* deltaproteobacteria (c_Deltaproteobacteria), and Vibrio butyricum spp. (g_Anaerostipes), which is consistent with the results of previous studies [16]. In addition, studies have reported some similarities between the intestinal flora of pregnant women with GDM and those with type 2 diabetes; the relative abundance of Desulfovibrio spp. in the intestinal flora of type 2 diabetic patients was significantly higher than that of controls [17]. Vibrio vulcanus and Vibrio vulcanus family both belong to Vibrio phylum and are sulfate-reducing bacteria [18] that break down short-chain fatty acids such as acetic acid and butyric acid in the intestine [19], leading to a decrease in the amount of short-chain fatty acids in the body, resulting in abnormalities in immune regulation and increased levels of inflammatory factors and serum glucose levels [16]. Hydrogen sulfide produced by Vibrio desulfuricans by reducing sulfate [20] can damage intestinal epithelial cells [21], impairing the function of the intestinal barrier and causing metabolic endotoxemia, which can lead to insulin resistance. In addition, hydrogen sulfide can also promote increased secretion of inflammatory factors [22], leading to chronic inflammatory states, causing insulin resistance, and ultimately leading to the development of metabolic diseases such as diabetes and obesity [23].

The main metabolite of Vibrio butyric acid is butyric acid, which as a short-chain fatty acid plays an important role in reducing the inflammatory response of the body, maintaining the function of the intestinal barrier, improving immunity, inhibiting the growth of tumor cells, and maintaining glucose homeostasis and energy metabolism [16]. Our results showed that the abundance of Vibrio butyricus genus, a genus that played a beneficial role in glucose regulation, was significantly higher in pregnant women with GDM than in healthy pregnant women. Therefore, we speculated that there may be a “self-defense mechanism” within the intestinal flora to regulate the body's glucose metabolism when it was disturbed. In other words, the abundance of intestinal flora that elevates blood glucose will increase when the body's glucose homeostasis is imbalanced. At the same time, the abundance of flora that is beneficial to lowering blood glucose will also increase to regulate blood glucose homeostasis.

The genus Akkermansia (g_Akkermansia) under the phylum Wartybacter, is a popular group of organisms that is currently widely studied in scientific research. Previous domestic studies have found that the relative abundance of Akkermansia spp. in the gut of pregnant women with GDM is significantly lower than that of healthy pregnant women [24]. Studies have also reported a significant reduction in the abundance of Akkermansia in the intestinal flora of obese and type 2 diabetic patients [25]. To date, its specific mechanisms in suppressing obesity and improving diabetes are not fully understood, while some of the pathways of action of Akkermansia have been identified. Akkermansia can reduce endotoxin absorption not only by activating TLR2, stimulating mucus secretion, increasing the thickness of the mucus layer, repairing the tight junctions of intestinal epithelial cells, and maintaining the integrity of the intestinal barrier [26] but also via reducing serum levels of IL10 and TGF*β* to reduce chronic inflammation in pancreatic islets and inhibiting the development of metabolic endotoxemia, thereby delaying the development of obesity and diabetes mellitus [27]. The mouse study showed that A. muciniphila could increase insulin secretion by promoting the expression of genes related to insulin secretion, thereby reducing the body's blood glucose level [28]. In addition, Depommier et al. found that supplementation with either live or pasteurized Akkermansia muciniphila improved intestinal barrier function, increased insulin sensitivity, and reduced plasma insulin and total cholesterol levels, thereby improving obesity [29]. In this study, we found that the simple superrecombination of the phylum Verrucomicrobia (p_Verrucomicrobia), the class Verrucomicrobiae (c_Verrucomicrobiae), the order Verrucomicrobiales (o_Verrucomicrobiales), the family Verrucomicrobiaceae (f_Verrucomicrobia), and the genus Akkermansia (g_ Akkermansia) was all significantly higher in relative abundance than the healthy pregnant women group. This result has been inconsistent with previous studies, a phenomenon that has raised the question of whether changes in the relative abundance of specific strains are the etiology of a disease or whether the organism was responding to it. It is necessary to consider the question of the causal relationship between gut flora and the development of metabolic diseases in humans.

In this study, we found that the proportion of the thick-walled phylum was reduced and the proportion of the mimic phylum increased in the GDM-only group compared to the normal pregnant group during late pregnancy. This result is consistent with the findings of Jang et al. [30], but contrary to the findings of Wilson et al. [31], who found an increase in the proportion of thick-walled phyla and a decrease in the proportion of Bacteroides and Actinobacteria in the gut flora of pregnant women with GDM. However, some studies have also found no significant differences in the intestinal flora between pregnant women with GDM and healthy pregnant women in late pregnancy [32].

To date, relatively few studies have been conducted on the changes in the intestinal flora of pregnant women with GDM and overweight women. In this study, the species composition and diversity of the intestinal flora of GDM, overweight, and normal pregnant women were compared and analyzed at two different stages of pregnancy: midtrimester and late trimester. The intestinal flora of newborns in each group was analyzed at birth to provide a reliable basis for further clinical studies. The factors such as dietary habits, exercise, and insulin use that could potentially affect the intestinal flora were not excluded from this study. The relatively small sample size in the study may result in some bias in the results. The study only analyzed the intestinal flora and did not compare the blood lipid index, serum insulin, and inflammatory factor levels of the pregnant women in each group.

To date, research on the role of intestinal flora in the development of overweight and GDM and the specific mechanisms is still in its early stages. We need to follow the frontiers of scientific research, continue to explore the mysteries, and strive to find strong evidence for the use of intestinal flora as a target for the prevention and treatment of obesity and GDM to contribute to the health of mothers and children.

## 5. Conclusion

Gut microbiota is strongly linked to obesity and gestational diabetes.

## Figures and Tables

**Figure 1:** Histogram of the degree of sequence annotation for each sample at each taxonomic level. The horizontal coordinate is the sample name, and the vertical coordinate indicates the ratio of the number of sequences annotated to that level to the total annotated data (sequence number percent). The top-down color order of the bars corresponds to the color order of the legends on the right. The highest value of 1 for each classification level means that 100% of the sequences were annotated at least at that level.

**Figure 2:** Relative distribution of phylum levels. The horizontal coordinate is the group name, the vertical coordinate (sequence number percent) indicates the ratio of the number of sequences annotated to that gate level to the total annotated data, and the top-down color order of the bars corresponds to the color order of the legends on the right. Sequences that are not annotated at the gate level are classified as unclassified. The legend shows up to 20 of the most dominant species, with the remaining species of lower relative abundance categorized as other shown in the figure. (a–c) indicate the relative distribution of gut flora at the phylum level for 24 weeks, 37 weeks, and neonates, respectively.

**Figure 3:** LDA histogram of intestinal flora LEfSe analysis for each group of pregnant women at 24 weeks.

**Figure 4:** LDA histogram of intestinal flora LEfSe analysis for each group of pregnant women at 37 weeks.

**Figure 5:** LDA histogram for LEfSe analysis of the intestinal flora of each group of neonates.

**Figure 6:** Common or endemic species Venn diagram.

**Figure 7:** PERMANOVA analysis based on Bray Curtis distance. The box line plot above shows grouping information horizontally, with the *n* value in brackets after each group name representing the number of comparisons between groups. The vertical is the distance between the samples compared. There were as many box plots as there were subgroups, and the above plots only showed the box plots plotted for all subgroups against the distance between samples from the first of these subgroups. (a) Represented the PERMANOVA analysis based on Bray Curtis distances between subgroups for 24 weeks of pregnant women; (b–d) represent the PERMANOVA analysis based on Bray Curtis distances between subgroups within the G_NO group, NG_O group, and NG_NO group, respectively. Curtis distance-based PERMANOVA analysis between groups within the G_NO group, NG_O group, and NG_NO group, respectively. Table 7 illustrates the detailed data for the box line plots. *P* < 0.05 inferred that there were significant differences in colony structure between groups.

**Figure 8:** Heat map of the interrelationships between microbial genus and clinical phenotypes at the genus level. Environmental factors were shown on the *x*-axis and species on the *y*-axis. The *R*-values (rank correlation) and *P* values were obtained by calculating the *R*-values, which were shown in different colors. *P* values less than 0.05 were marked with an ∗. (b) The legend on the left showed the color intervals for the different *R*-values, while the color bar on the right indicated the phylum to which the species belongs.

**Table 1:** The details of main experimental reagents.

Reagent name	Type	Company	Country
DNA Extraction Kits	OMEGA-Soil DNA Kit	Omega Bio-Tek	USA
2% agarose gels	Biowest agarose	Biowest	Spain
FastPfu Polymerase	FastPfu Polymerase	TransGen	China
AxyPrep DNA Gel Extraction Kit	Axygen Biosciences	Axygen	USA
Illumina MiSeq platform	TruSeq™ DNA Sample Prep Kit	Illumina	USA

**Table 2:** The details of main experimental instruments.

Instrument	Type	Company	Country
Pipettes	Eppendorf N13462C	Eppendorf	Germany
Micro centrifuge	ABSON MiFly-6	Aibensen Scientific Instrument Co., Ltd	Hefei, China
Compact centrifuge	Eppendorf 5430 R	Eppendorf	Germany
Ultramicro-spectrophotometer	NanoDrop2000	Thermo Fisher Scientific	USA
Electrophoresis instrument	DYY-6C	Beijing Liuyi Instrument Factory	China
PCR instrument	ABI GeneAmp® 9700	ABI	USA
MiSeq sequencer	Illumina MiSeq	Illumina	USA
Vortex mixers	QL-901	Kylin-Bell Lab Instruments Co., Ltd.	Haimen, China
Crushing and grinding instrument	TL-48R	Wonbio Biotechnology Co., Ltd.	Shanghai, China

**Table 3:** Number of feces collected.

	NG_NO	G_NO	NG_O	G_O	Total (n)
24-week gestation	15	6	7	4	32
37-week gestation	15	4	7	3	29
Neonates	12	2	2	2	18
In total (*n*)	42	12	16	9	79

**Table 4:** PCR amplification of 16s rRNA V3-V4 variable region.

Sequencing region	Primer name	Primer sequence
338F_806R	338F	ACTCCTACGGGAGGCAGCAG
	806R	GGACTACHVGGGTWTCTAAT

**Table 5:** PCR amplification system.

Reagents	Dose
5 × FastPfu buffer	4 *μ*l
2.5 mM dNTPs	2 *μ*l
Forward primer (5 *μ*M)	0.8 *μ*l
Reverse primer (5 *μ*M)	0.8 *μ*l
FastPfu Polymerase	0.4 *μ*l
BSA	0.2 *μ*l
Template DNA	10 ng

**Table 6:** PCR amplification reaction procedure.

Temperature (°C)	Lasting time	Cycle (*n*)
95	3 min	1
95	30 s	27
55	30 s	27
72	45 s	27
72	10 min	1

**Table 7:** PERMANOVA analysis based on Bray Curtis distance.

Group 1	Group 2	*F* value	*P* value
G_NO_24W	G_O_24W	0.878325	0.660
	NG_O_24W	1.204852	0.125
	NG_NO_24W	1.081780	0.291
	G_NO_37W	0.780509	0.732
	G_NO_newborn	3.755146	0.039
G_O_24W	NG_O_24W	0.475199	1.000
	NG_NO_24W	1.160615	0.222
NG_O_24W	NG_NO_24W	1.502780	0.020
	NG_0_37W	0.534072	0.972
	NG_0_newborn	2.603314	0.022
NG_NO_24W	NG_NO_37W	0.466387	0.998
	NG_NO_newborn	25.629649	0.001
G_NO_37W	G_NO_newborn	4.481362	0.065
NG_0_37W	NG_0_newborn	3.480097	0.027
NG_NO_37W	NG_NO_newborn	23.104469	0.001

## Data Availability

The datasets used and analyzed during the current study are available from the corresponding author upon reasonable request.
